# PTIP Inhibits Cell Invasion in Esophageal Squamous Cell Carcinoma *via* Modulation of EphA2 Expression

This article has been retracted.

**DOI:** 10.3389/fonc.2021.629916

**Published:** 2021-03-23

**Authors:** Xiao Han, Yaning Zhu, Li Shen, Yu Zhou, Liqun Pang, Wubi Zhou, Hao Gu, Kairong Han, Yijun Yang, Chao Jiang, Jun Xie, Chengwan Zhang, Lianshu Ding

**Affiliations:** ^1^ Department of Central Laboratory, The Affiliated Huaian No. 1 People’s Hospital of Nanjing Medical University, Huai’an, China; ^2^ Department of Pathology, The Affiliated Huaian No. 1 People’s Hospital of Nanjing Medical University, Huai’an, China; ^3^ Department of Hematology, The Affiliated Huaian No. 1 People’s Hospital of Nanjing Medical University, Huai’an, China; ^4^ Department of Medical Oncology, The Affiliated Huaian No. 1 People’s Hospital of Nanjing Medical University, Huai’an, Jiangsu, China; ^5^ Department of General Surgery, The Affiliated Huaian No. 1 People’s Hospital of Nanjing Medical University, Huai’an, China; ^6^ Department of Obstetrics and Gynecology, The Affiliated Huaian No. 1 People’s Hospital of Nanjing Medical University, Huai’an, China; ^7^ Department of Clinical Laboratory, Xuyi People’s Hospital, Huai’an, China; ^8^ Department of Neurosurgery, The Affiliated Huaian No. 1 People’s Hospital of Nanjing Medical University, Huai’an, China

**Keywords:** esophageal squamous cell carcinoma, PTIP, EphA2, Fosl2, invasion

## Abstract

Esophageal squamous cell carcinoma (ESCC) is a highly aggressive malignancy and treatment failure is largely due to metastasis and invasion. Aberrant tumor cell adhesion is often associated with tumor progression and metastasis. However, the exact details of cell adhesion in ESCC progression have yet to be determined. In our study, the clinical relevance of Pax2 transactivation domain-interacting protein (PTIP/PAXIP1) was analyzed by immunohistochemistry of ESCC tissues. We found that low expression of PTIP was associated with lymph node metastasis in ESCC, and loss-of-function approaches showed that depletion of PTIP promoted ESCC cell migration and invasion both *in vitro* and *in vivo*. Analysis integrating RNA-seq and ChIP-seq data revealed that PTIP directly regulated ephrin type-A receptor 2 (EphA2) expression in ESCC cells. Moreover, PTIP inhibited EphA2 expression by competing with Fosl2, which attenuated the invasion ability of ESCC cells. These results collectively suggest that PTIP regulates ESCC invasion through modulation of EphA2 expression and hence presents a potential therapeutic target for its treatment.

## Introduction

Esophageal cancer, a highly aggressive malignancy, globally ranks seventh in the incidence of cancer cases and sixth as the leading cause of cancer-related deaths. Moreover, in 2018, the number of new esophageal cancer cases and deaths worldwide was about 572000 and 509000, respectively (1). According to histopathological analysis, esophageal carcinoma can be classified as two main types: esophageal squamous cell carcinoma (ESCC) and esophageal adenocarcinoma (EAC) (2). ESCC is the predominant subtype of esophageal cancer in China, accounting for 90% of esophageal carcinomas (3). Approximately 50% of patients when diagnosed with ESCC already have distant metastases and more than one-third develop distant metastases following surgery or radiotherapy (4, 5). In addition, most distant metastases of ESCC involve the distant lymph nodes (5). Therefore, dissecting the mechanisms underlying esophageal cancer invasion and metastasis is fundamental for the development of effective therapeutic strategies to improve patients’ outcomes.

Tumor invasion and metastasis are complex processes based on angiogenesis and the weakening of tumor cell adhesion, that involve multiple stages, genes, and the accumulation of different factors (6). Receptor tyrosine kinases (RTKs) function as key regulators of signal transduction pathways that control cell proliferation, survival and migration in the progression of malignant solid tumors. EphA2 belongs to the Eph family, the largest family of membrane-bound receptor tyrosine kinases (7). Previous works show that EphA2 has dual roles in both promoting and inhibiting cancer cell metastatic progression (8, 9). In breast cancer, ligand-dependent EphA2 signaling inhibits proliferation and invasiveness, whereas ligand-independent manner promotes tumor malignancy through EphA2 phosphorylation at serine-897 (9, 10). Recent study has shown that EphA2 is highly expressed and associated with poor degree of tumor differentiation and lymph node metastasis in ESCC (11). However, how EphA2 is modulated in ESCC remains unclear.

PTIP (Pax2 transactivation domain-interacting protein) is a nuclear protein containing six BRCT domains and is an essential component of histone H3K4 methyltransferase complexes that are associated with gene activation (12), DNA repair (13, 14), embryonic vascular development (15), and embryonic stem cell pluripotency (16). In addition, PTIP can interact with the Pax family of transcription regulators and inhibit the transactivation of the glucagon promoter in pancreatic cells (17). Recent studies have shown that low PTIP is associate with more aggressive tumor phenotypes in breast cancer (18). Results from a meta-analysis analysis also found that downregulation of PTIP was associated with poor prognosis in ovarian cancer (19). These data suggest that PTIP can inhibit tumor progression.

In this study, we examined the role of PTIP in ESCC by analyzing the expression characteristics of PTIP in esophageal tumor tissues. The biological function and underlying molecular mechanisms of PTIP in ESCC invasion were also investigated. Here we found that low expression of PTIP was positively associated with ESCC tissue lymph node metastasis. Moreover, we demonstrated that PTIP participates in ESCC invasion and metastasis *via* suppressing the expression of EphA2, a crucial factor involved in tumor cell adhesion.

## Materials and Methods

### Patient Information and Tissue Samples

Eighty-seven patients with ESCC underwent surgery with curative intent at the Affiliated Huaian No.1 People’s Hospital of Nanjing Medical University (Huai’an, China). Those with confirmed or suspected lymph node metastasis received regional lymph node dissection. All patients provided written informed consent. The study protocol was approved by the Huaian No.1 People’s Hospitals’ Ethics Committee (No. YX-2020-162-01). The resected specimens were fixed in 10% formaldehyde solution and embedded in paraffin. The tumor stage was classified according to the 5th edition of the TNM classification of the International Union against Cancer (UICC).

### Cell Culture

HEK293T cells and human ESCC cell lines, including TE1 and KYSE-150 were obtained from the Chinese Type Culture Collection (Shanghai, China) and cultured in Dulbecco’s modified Eagle’s medium (DMEM, Gibico, C11995500BT, Beijing, China) supplemented with 10% fetal bovine serum (FBS, AusgeneX, FBSSA500-S, QLD, Australia) and 1% penicillin/streptomycin (Gibico, 15140-122, USA) at 37°C in a humidified incubator with 5% CO_2_. All cells were tested negative for mycoplasma.

### Mouse Experiments

Female BALB/c nude mice (4–5 weeks old) were purchased from Nanjing Medical University and housed in a specific-pathogen-free barrier facility with free access to food and water. All animal experiments were approved by the Animal Experimentation Ethics Committee of Huai’an First People’s Hospital. KYSE-150 cells (1×10^6^) were infected with scrambled shRNA (shCtrl) or shPTIP#1 lentivirus containing a constitutively expressed luciferase reporter for 72 hours. Each group of cells were injected into the lateral tail vein of nude mice (n=8). The transplanted animals were monitored *in vivo* every week by bioluminescent imaging. Anesthetized mice were injected intraperitoneally with D-Luciferin (150 mg/kg, D1007, US Everbright, China) and were imaged with 2 min acquisition time using an In-Vivo FX PRO (BRUKER, NY, USA) imaging system, 10 min after injection. The bioluminescence intensity of the captured images were quantitated using Bruker MI SE acquisition and analysis software (BRUKER). Four weeks later, mice were euthanized, and lung tissue sections were stained with Hematoxylin-Eosin (H&E) for histopathological analysis.

### Vector Construction

Lentiviral vectors harboring short hairpin RNA (shRNA) targeting PTIP (shPTIP), Fosl2 (shFosl2) and EphA2 (shEphA2) were synthesized by Genscript (Nanjing, China). cDNAs encoding PTIP were cloned into the expression vector pLenti-EFs-BSD with a blasticidin-resistant gene for N-terminal tagging of MYC epitope (PTIP-MYC) or FLAG epitope (PTIP-FLAG). Lentiviral luciferase-expressing vectors pLVshRNA-Luci(2A)-puro-shScrambled and pLVshRNA-Luci(2A)-puro-shPTIP were constructed by cloning shScrambled and shPTIP into pLVshRNA-Luci(2A)-puro vector (Inovogen, Beijing, China), respectively. The primer sequences used for plasmid construction are listed in **Table 1**.

**Table 1:** Primers used for plasmid construction.

Primer	Sequence (5ʹ-3ʹ)
shPTIP-1-forward	GATCGGGGCAGGAAGACAGATATAATAACGAATTATTATATCTGTCTTCCTGCTTTTTC
shPTIP-1-reverse	AATTGAAAAAGCAGGAAGACAGATATAATAATTCGTTATTATATCTGTCTTCCTGCCCC
shPTIP-2- forward	GATCGGGGCAGCAACACAGTCCTCATCTCGAAAGATGAGGACTGTGTTGCTGCTTTTTC
shPTIP-2- reverse	AATTGAAAAAGCAGCAACACAGTCCTCATCTTTCGAGATGAGGACTGTGTTGCTGCCCC
shFosl2-1- forward	GATCGGGGGATTATCCCGGGAACTTTGACGAATCAAAGTTCCCGGGATAATCCTTTTTC
shFosl2-1- reverse	AATTGAAAAAGGATTATCCCGGGAACTTTGATTCGTCAAAGTTCCCGGGATAATCCCCC
shFosl2-2- forward	GATCGGGGATCATGTACCAGGATTATCCCGAAGGATAATCCTGGTACATGATCTTTTTC
shFosl2-2- reverse	AATTGAAAAAGATCATGTACCAGGATTATCCTTCGGGATAATCCTGGTACATGATCCCC
PTIP- forward	GGATCTATTTCCGGTGAATTCCATGTCGGACCAGGCGC
PTIP- reverse	GGAGGGAGAGGGGCGGGATCCCCAGATCCTCTTCTGAGATGAGTTTCTG
shScrambled- forward	GATCGGGTTCTCCGAACGTGTCACGTTTCCGAAGAAACGTGACACGTTCGGAGAATTTTTC
shScrambled- reverse	AATTGAAAAATTCTCCGAACGTGTCACGTTTCTTCGGAAACGTGACACGTTCGGAGAACCC
shEphA2-1-forward	GATCGGGGCATCTTCCTAGTGCCCTACTCGAAAGTAGGGCACTAGGAAGATGCTTTTTC
shEphA2-1- reverse	AATTGAAAAAGCATCTTCCTAGTGCCCTACTTTCGAGTAGGGCACTAGGAAGATGCCCC
shEphA2-2-forward	GATCGGGGCTCCTCTTTATACCTCTAGACGAATCTAGAGGTATAAAGAGGAGCTTTTTC
shEphA2-2- reverse	AATTGAAAAAGCTCCTCTTTATACCTCTAGATTCGTCTAGAGGTATAAAGAGGAGCCCC

### Real-Time Quantitative Polymerase Chain Reaction (RT-qPCR)

Total RNA in ESCC cells was extracted using RNeasy Kits (Qiagen, 74104, Hilden, Germany) according to the manufacturer’s instructions. Primescript RT-reagent kit (Takara, RR047A, Shiga, Japan) was used to synthesize cDNA. SYBR Premix Ex Taq (Takara, Dalian, China) was used for qPCR. qPCR analysis was performed using LightCycler 480 system (Roche, Basel, Switzerland) and the data were analyzed by the ΔΔCt method with normalization to β-actin. The primer sequences used for real-time PCR are listed in **Table 2**.

**Table 2:** Primers used for Real-time PCR.

Primer	Sequence (5ʹ-3ʹ)
PTIP-RT-forward	CCAGCTGTACGGACACTGAGG
PTIP-RT-reverse	TTGTATGTCCCTGCTGGCTGT
EphA2- RT-forward	TGGCTCACACACCCGTATG
EphA2- RT- reverse	GTCGCCAGACATCACGTTG
TACSTD2- RT-forward	CGGCAGAACACGTCTCAGAAG
TACSTD2- RT-reverse	CCTTGATGTCCCTCTCGAAGTAG
GPRC5A - RT- forward	ATGGCTACAACAGTCCCTGAT
GPRC5A - RT- reverse	CCACCGTTTCTAGGACGATGC
β-actin- RT-forward	AAGACCTGTACACCAACACAG
β-actin- RT-reverse	AGGGCAGTGATCTCCTTCT
BML-RT-forward	CAGACTCCGAAGGAAGTTGTATG
BML-RT-reverse	TTTGGGGTGGTGTAACAAATGAT
P53-RT-forward	CAGCACATGACGGAGGTTGT
P53-RT-reverse	TCATCCAAATACTCCACACGC

### Western Blot

Proteins were isolated from human ESCC cells using lysis buffer (2% SDS, 62.5 mM Tris pH 6.8, 10% glycerol, 5% β-mercaptoethanol) and supplemented with an EDTA-free protease inhibitor cocktail (Roche, 4693132001, MO, USA), phosphatase inhibitor cocktail (MCE, HY-K0021, NJ, USA), and PMSF (MCE, HY-B0496, NJ, USA). SDS-PAGE was used to separate the proteins with different molecular weights (45 min, 200 V) (Bio-Rad Laboratories) and then transferred onto PVDF membranes (LC2002, Invitrogen, CA, USA) using a wet blotting system (70 min, 250 mA) (BioRad Laboratories). Membranes were blocked with 5% non-fat milk in TBST and then incubated with primary antibodies, followed by the appropriate secondary antibody.

The antibodies used in this study are listed as follows: PTIP (1:2000, 130kDa, A300-370A, BETHYL, USA), EphA2 (1:1000, 108 kDa, AF5238, Affinity Biosciences, USA), pS897-EphA2(1:1000, 125 kDa, 6347S, CST, USA), pY588-EphA2(1:1000, 125 kDa, 12677S, CST, USA), YY1 (1:1000, 70kDa, 22156-1-AP, Proteintech, USA), MYC (1:1000, 16286-1-AP, Proteintech, IL, USA), FLAG (1µg/µL, T0003, Proteintech, IL, USA), Fosl2 (1:1000, 35 kDa, A2729, ABclonal, USA), GAPDH (1:2000, 36 kDa, AP0063, Bioworld, Nanjing, China), β-actin (1:2000, 42 kDa, 20536-1-AP, Proteintech, IL, USA).

Proteins were detected using a chemiluminescence reagent (WesternBright peroxide, Advansta, CA, USA) in a ChemiDoc XRS+ System (Bio-Rad, CA, USA).

### Immunohistochemistry

Paraffin-embedded blocks from human specimens or mouse xenografts were sectioned into 4-μm thick slices and positioned on pre-coated slides. The unstained slides were deparaffinized, rehydrated, and incubated with fresh 0.3% H_2_O_2_ in methanol for 30 min at about 25°C. Thereafter, antigen retrieval was performed in 10 mM citrate buffer by heating the samples to 121°C. Tissue sections were then blocked for 30 min with 5% horse serum in PBST and incubated with the primary antibody at 4°C overnight, washed in PBS, and incubated with secondary antibody for 2 h at room temperature. Immunoreactivity was visualized by DAB chromogen followed by hematoxylin counterstain. Two pathologists scored the staining of PTIP and EphA2 independently, then a multiplicative Quick-score (Q-score) was calculated by multiplying the percentage of positive cells by the intensity of the staining. Ten sections were collected randomly, and the average Q-score was calculated for each section.

### RNA-Seq Analysis

Transcriptome analyses were performed to compare the control TE1 with PTIP-depleted cells. This same methodology was applied to compare non-invasive with invasive tumor biopsies from ESCC patients. cDNA libraries were generated using NEB Next Ultra Directional RNA Library Prep Kit (NEB) following the manufacturer’s instructions, and then sequenced using the Illumina sequencing technology on an Illumina Novaseq 6000 at LC Bio (Zhejiang, China) according to the manufacturer’s instructions. Differential expression analysis of the two groups was performed using the ballgown R package (20). The resulting *P*-values were adjusted using Benjamini and Hochberg’s approaches to control the false discovery rate. Genes with an adjusted *P*-value <0.05 were considered to be differentially expressed. The clusterProfiler R package was used to detect the statistical enrichment of differentially expressed genes in Gene Ontology (GO).

### Chromatin Immunoprecipitation Sequencing (ChIP-Seq) Analysis

ChIP-seq experiments were performed on TE1 cells overexpressed with MYC-tagged PTIP. For histone ChIP–seq, cells were fixed in 1% formaldehyde (FA, Thermo Fisher Scientific, 28906) for 10 min at room temperature. The reaction was stopped by the addition of glycine (0.125 M, Sigma), and the cells were washed in ice-cold PBS. Cells were sonicated using a Bioruptor sonicator (Diagenode) until 200–500 bp DNA fragments were obtained. Further procedures were performed according to Richard A Young’s protocol (21). DNA libraries were sequenced on an Illumina HiSeq platform (Novogene, Beijing, China). The sequencing data were mapped to the hg38 genome, and peak calling was performed using Model-based analysis of ChIP-Seq (MACS) version 2.1.1 with default parameters to obtain primary binding regions. The pie plot and heatmap of ChIP binding the TSS regions were generated using the ChIPseeker R package (22). Motif discovery was performed using HOMER. ChIP-Seq datasets were subsequently visualized using the IGV software.

### Chromatin Immunoprecipitation Quantitative Real-Time PCR (ChIP-qPCR)

ChIP assays were performed with a Millipore ChIP kit according to the manufacturer’s protocol (21). Briefly, 3×10^7^ cells were collected, fixed, and sonicated with a Bioruptor sonicator (Diagenode) to generate DNA fragments of approximately 500 bp in length. Chromatin immunoprecipitates for proteins were amplified by quantitative PCR, normalized to input, and calculated as percentages of inputs. Fold enrichment levels indicate fold changes over the negative control immunoglobulin G (IgG). The PCR primer sequences are listed in **Table 3**.

**Table 3:** Primers used for ChIP-qPCR.

Primer	Sequence (5ʹ-3ʹ)
EphA2-F forward	GCCCTTATCGTGACGCAAGT
EphA2-F reverse	CCCTAGGTGAATTGCCACCA
EphA2-NC-forward	CAGCAGGCAGTGGGATGAG
EphA2-NC- reverse	TCCCACAGCTAGGAGGTGACA

### Transwell Assay

Cells (4×10^4^/well) resuspended in serum-free DMEM were added to the upper transwell chambers coated with matrigel. DMEM with 10% FBS was added to the lower chambers. After 48 h of incubation at 37°C, cells remaining in the upper chamber were wiped with cotton buds, whereas cells that had invaded the lower chamber were fixed with 10% methanol and stained with 0.1% crystal violet. Images were captured under a microscope. Each transwell assay was conducted in duplicate and repeated 3 times. The rate of invasion was measured using an ImageJ analysis system (version 1.8.0; National Institutes of Health, Bethesda, MD, USA).

### Wound Healing Assay

Cells (6×10^5^/well) were seeded into a 6-well culture plate. The next day, when the cells were almost 80% confluent, a 10 µL pipette tip was used to scratch artificial linear wounds in the monolayer. Cells were washed 3 times with PBS and cultured in serum-free DMEM at 37°C. The width of the scratch gap was monitored by microscopy and photographed at 0 h and 12 h. The cell migration rate was quantified according to the original width of the wound and the width after cell migration. The ImageJ analysis system was used to analyze the rate.

### Apoptosis Assay

Analyses were performed using YF647A-AnnexinV/PI apoptosis detection kit (Y6026, US EVERBRIGHT, Suzhou, China) according to the manufacturer’s protocol. Briefly, ESCC cells were seeded into 6-well plates with 5 × 10^5^. After the cell density reached 80∼90%, cells were then harvested and washed with PBS for three times before addition of 500 μL binding buffer, 5 μL YF647A-AnnexinV and 5 μL PI solution to the cell pellet for 15 min at room temperature in the dark before flow cytometric analysis to detect early apoptotic cells (Annexin-V positive and PI-negative) and late apoptotic cells (Annexin-V and PI double positive)(Beckman Coulter, USA).

### Cell-Matrix Adhesion Assay

ESCC cells were seeded at a density of 2×10^5^ per ml (100 µl per well) in 96-well plates coated with Collagen I (40 µg/ml; Corning, NY, USA). Following 1 h incubation at 37°C in an incubator containing 5% CO2, the cells were washed with PBS to remove non-adherent cells. A total of 10 µl CCK8 (Dojindo, CK04, Japan) was added to each well. Following 1 h of additional incubation, absorbance values were determined using Hidex Sense instrument (Hidex, Finland) at a wavelength of 450 nm. The percentage of adhesive cells was calculated according to the following formula: Percentage of adhesion= [(optical density (OD) 450 of PTIP knockdown cells-Blank)/(OD450 of Ctrl cells-Blank)]x100%. Three independent experiments were performed in triplicate.

### Immunofluorescence by Confocal Microscopy

ESCC cells were cultured on glass coverslips, fixed with 4% paraformaldehyde in PBS for 20 min, and subsequently permeabilized with 0.5% Triton X-100 for 10 min. Cell were incubated with phalloidin (YP0063, US EVERBRIGHT, Suzhou, China) for 20 min at room temperature. After three washes with PBS, cells were mounted with Aqueous Mounting Medium containing 4’,6-diamidino-2-phenylindole (DAPI, Beyotime, C1005, Shanghai, China) and visualized with a confocal microscope.

### Statistical Analysis

SPSS software version 19.0 (IBM Corp., Armonk, New York, US) and GraphPad Prism v6 (GraphPad Software, Inc., San Diego, California, US) were used for all statistical analyses. Data were first evaluated for normal distribution using the Shapiro-Wilk method and homogeneity of variance with the Levene method. Pairwise comparisons of normally distributed data were analyzed using Student’s t test or for multigroup comparisons, one-way analysis of variance (ANOVA) with *post hoc* Tukey’s test. Data not meeting normal distribution/homogeneity of variance were compared using Kruskal-Wallis and Mann-Whitney non-parametric tests. Data are presented as the mean ± SEM (error bars). *P* < 0.05 (*), *P* < 0.01 (**), and *P* < 0.001 (***) denote statistically significant changes.

## Results

### PTIP Expression Negatively Correlates With Lymph Node Metastasis in ESCC

To identify metastatic genes during ESCC progression, we used an RNA-seq-based approach to compare the transcription profile differences between non-invasive and invasive tumor biopsies from ESCC patients. Overall, 776 genes were differentially expressed. Of these, 435 genes were upregulated in invasive tumor samples while 341 genes were downregulated (**Figure 1A**). We conducted functional enrichment analysis using online tool Metascape and obtained significant enrichment CORUM (the comprehensive resource of mammalian protein complexes) gene set and Gene Ontology (GO) terms (three terms: Biological Process: BP, Cellular Component: CC and Molecular Function: MF). We had 2 significant CORUM gene set, 330 significant GO: BP terms, 28 significant GO : CC terms and 58 significant GO : MF terms. The top CORUM gene set from the functional enrichment analysis of DEGs is “PTIP-DNA damage response complex” (**Figures 1B, C**). Of this set of genes, three were downregulated in patients with lymph node metastasis, including BLM, TP53 and PTIP. These genes were further investigated by RT-qPCR. The results shown that the most significantly changed gene was PTIP (**Figure 1D**).

**Figure 1:** PTIP expression negatively correlates with lymph node metastasis in ESCC. **(A)** Volcano plot showing differentially expressed genes between tumor biopsies with and without lymph node metastasis using RNA-seq. Volcano plot shows the log2 fold change (x-axis) and significance (−log10*adjusted *P*-value; y-axis) with significantly downregulated and upregulated genes shown in blue and red, respectively (adjust *P* < 0.01 and |log2Foldchange| > 0.9). **(B)** GO enrichment of differentially expressed genes from **(A)**. **(C)** Functional enrichment analysis of differentially expressed genes from **(B)** using CORUM gene set. **(D)** quantitative RT-PCR analysis of genes that downregulated in lymph node metastasis positive ESCC samples. Unpaired, two-tailed Student’s t-test; *P < 0.05; ***P < 0.001; n.s., not significant. **(E)** IHC score for PTIP in ESCC tumor sections. Unpaired, two-tailed Student’s t-test; **P < 0.01. **(F)** Representative IHC images for PTIP in ESCC tumor sections. Low PTIP and high PTIP groups were divided based on the PTIP immunostaining intensity scores mentioned in method. Cut off for high and low PTIP expression in ESCC was defined < or > 11. Percentage of invasion and non-invasion in ESCC groups is depicted in **Table 4**.

We next analyzed the correlation between PTIP expression and the clinicopathological parameters in tissues from 79 ESCC patients. The expression of PTIP varies greatly in ESCC tissues (**Figure 1E**). Based on the PTIP immunostaining intensity scores mentioned in the Methods section, the cohort of 79 ESCC patients were divided into low PTIP and high PTIP groups. We found a statistically significant negative correlation between PTIP nuclear expression in ESCC and lymph node status (*P* = 0.0399; **Tables 4**, **S1** and **Figure 1F**). PTIP staining intensity was higher in lymph node metastasis–negative samples when compared with metastasis-positive samples. When taken in context with our PTIP RNAi sequencing data, our findings indicate that PTIP was reduced in more aggressive ESCC phenotypes.

**Table 4:** Summary of clinical and histopathological characteristics of the 79 esophageal squamous cell carcinoma patients.

Variables	All cases(N=79; %)	PTIP		*P*-values
		Low (n = 25; %)	High(n = 54; %)	
Gender				0.5995/0.4599
Male	55(69.6)	16(20.3)	39(49.4)	
Female	24(30.4)	9(11.4)	15(19.0)	
Age(year)				0.3323/0.2452
<65	36(45.6)	9(11.4)	27(34.2)	
>=65	43(54.4)	16(20.3)	27(34.2)	
Size(cm)				0.3845/0.3402
<5	62(78.5)	18(22.8)	44(55.7)	
>=5	17(21.5)	7(8.9)	10(12.7)	
Grade				0.973
Poor	27(34.2)	7(8.9)	20(25.3)	
Moderate	34(43.0)	14(17.7)	20(25.3)	
Well	18(22.8)	4(5.1)	14(17.7)	
TNM Stage				0.4338/0.4015
I-II	24(30.4)	6(7.6)	18(22.8)	
III-IV	55(69.6)	19(24.1)	36(45.5)	
Lymph node status				0.0399/0.0231*
0	52(65.8)	12(15.2)	40(50.6)	
>=1	27(34.2)	13(16.5)	14(17.7)	
Distant metastasis				
M0	79(100)	25(31.6)	54(68.4)	
M1	0(0)	0(0)	0(0)	

The numbers in parentheses indicate the percentages of tumors with a special clinical or pathologic feature for a given PTIP subtype.

The differences between rates were tested by χ2 or Fisher exact tests, if appropriate. *Statistically significant.

### Knockdown of PTIP Promotes ESCC Cell Invasion and Migration

To investigate the function of PTIP in ESCC, we silenced PTIP in TE1 and KYSE-150 cell lines using shRNA lentivirus. PTIP knockdown substantially promoted the invasion abilities of TE1 and KYSE-150 cells (**Figures 2A–F**). Furthermore, the wound healing assay demonstrated that suppression of PTIP resulted in a higher scratch closure rate compared with control groups (**Figures 2G–J**). To exclude the effect of cell apoptosis on cell migration, we conducted an apoptosis assay in ESCC cells using Annexin V and PI staining. Flow cytometry revealed that there were no remarkable differences in apoptosis rate between shPTIP and shCtrl cells (**Figures S1a, b**). Moreover, the EC-matrix adhesion ability and cell morphology of ESCC cell lines were determined by cell-matrix adhesion assay and phalloidin staining, respectively. No significant differences were observed between shPTIP and shCtrl cells (**Figures S1c, d**). Furthermore, we checked the effect of PTIP overexpression in ESCC cells, observing that transformed cells did not significantly inhibit cell invasion (**Figures S2a-f**). This may be duo to endogenously-expressed basal level of PTIP is high enough to suppress ESCC cell invasion. Collectively, these findings indicate that PTIP is important for the invasion and migration of ESCC cells.

**Figure 2:** Effects of PTIP on ESCC cell invasion and migration. **(A, B)** Knockdown efficiency of two independent shRNAs targeting PTIP in TE1 **(A)** and KYSE-150**(B)** cells as determined by qRT-PCR and Western blot. **(C–F)** The effect of PTIP knockdown on the invasiveness of TE1 **(C, D)** and KYSE-150**(E, F)** cells. For invasion assay, six different microscopic fields (magnification, ×10) from at least three independent experiments were examined; Relative intensities of the fields were measured (n ≥3). Representative images and statistical plots are shown; Mean ± s.d. are given for three independent experiments. One-way ANOVA; *P < 0.05,**P < 0.01, ***P <0.001. **(G–J)** Wound healing assay was performed to determine the cell migration in TE1 **(G, H)** and KYSE-150 **(I, J)** cells. Representative images and statistical plots are shown; Mean ± s.d. are given for three independent experiments. One-way ANOVA; *P < 0.05,**P < 0.01.

Further, to determine the role of PTIP in ESCC invasion *in vivo*, we treated KYSE-150 cells with shScrambled-Luc (control) or shPTIP#1-Luc-containing viruses, and subsequently delivered these 2 groups of cells into mice by tail vein injection. *In vivo* imaging analysis demonstrated that mice injected with shPTIP-Luc-treated KYSE-150 cells had stronger luciferase signals than those injected with shScrambled-Luc treated KYSE-150 cells (**Figure 3A**). In particular, there was a significant difference in the luciferase signal between shScrambled-Luc group and shPTIP group at 4th week (**Figure 3B**). Metastatic tumors in bioluminescence-positive tissues were further confirmed by H&E staining (**Figure 3C**). These results suggest that depletion of PTIP promotes invasiveness of ESCC cells *in vivo*.

**Figure 3:** PTIP inhibits ESCC cell invasion and migration *in vivo.* ***(*A, B*)*** The effect of PTIP knockdown on tumor growth and metastasis in a mouse model based on tail vein injection. KYSE-150 cells were infected with Scrambled shRNA (shCtrl) or shPTIP#1 lentivirus containing a constitutively expressed luciferase reporter. Then, shScrambled-treated or shPTIP cells were injected into mice *via* tail veins(n=8), and lung metastases in the two groups were evaluated by an *in vivo* imaging system(In-Vivo FX PRO). The luciferase signals were compared between the shCtrl group and the shPTIP group. Unpaired, two-tailed Student’s t-test; *P < 0.05. **(C)** Metastatic lesions in lungs from mice at the 4^th^ week were analyzed by H&E staining. Overall staining patterns were shown at low magnification (original magnification ×5) as a composite figure and zoomed views (original magnification ×20) of the indicated areas (box).

### PTIP Attenuates EphA2 Gene Expression in ESCC Cells

A comparative analysis of the transcriptomes between the two groups of ESCC cells (shScrambled vs. shPTIP) was performed to understand the mechanism by which PTIP attenuates ESCC invasiveness. A total of 6005 differentially expressed genes (DEGs) were identified, of which 3076 were upregulated and 2929 downregulated (**Figure 4A**). GO enrichment analysis was performed for the DEGs to investigate the biological functions of these genes. The top 20 GO biological processes based on *P*-value are listed in particular (**Figure 4B**), the cell-cell adhesion processes were significantly changed after depletion of PTIP compared to control cells (**Table S2**).

**Figure 4:** Analysis of the differentially expressed genes(DEGs) and PTIP binding sites. **(A)** The differentially expressed genes between PTIP knockdown(shPTIP) and control (shScrambled) group were identified by RNA-seq analysis. Volcano plot shows the log2 fold change (x-axis) and significance (−log10 * adjusted p-value; y-axis) with significantly downregulated and upregulated genes shown in blue and red, respectively (adjust *P* < 0.01 and |log2Foldchange| < 1). **(B)** Gene ontology (GO) analysis for enrichment of the DEGs based on the results from **(A)** RNA sequencing. **(C)** Western blot verification of MYC tagged PTIP over-expression efficiency in TE1 cells. **(D–F)** PTIP binding sites and target genes were identificated by chromatin immunoprecipitation (ChIP)-Seq using MYC tag antibody in MYC tagged PTIP ESCC cell line. Pie charts showing the distribution of PTIP-binding sites in the genome. The percentage of binding sites are indicated in parentheses. The graphs were generated using the ChIPseeker, Deeptools and GOplot package in R. Binding profile around the transcription start site (TSS) of PTIP **(E)**. Mean read coverage is plotted (y-axis) against a sliding window around the TSS (x-axis). TES, transcription end site; TSS, transcription start site. Enrichment of biological process terms among PTIP target genes**(F)**. **(G)** Venn diagram showing the overlapping genes identified by RNA-Seq data and ChIP-Seq data. **(H)** Enrichment of biological process terms among the 38 overlapping genes. **(I)** qRT-PCR analysis of three potentially PTIP directly regulated cell-cell adhesion genes. Representative images and statistical plots are shown; Mean ± s.d. are given for three independent experiments. One-way ANOVA; **P < 0.01.

To further investigate the direct target of PTIP in ESCC cells, we used ChIP-Seq with a Myc tag antibody in ESCC cells overexpressing Myc-tagged PTIP (**Figure 4C**). We documented 8439 PTIP-binding sites, corresponding to 126 genes. Further analysis revealed that more than 57% of the binding sites were found at the promoter and transcription start site (TSS) regions of annotated genes (**Figure 4D**), with the peak regions located at −3,000 to +3,000 bp from the TSS (**Figure 4E**), supporting the hypothesis that PTIP may function as a transcriptional co-factor. Among the PTIP target genes, genes assigned to the terms “Transcription, DNA-templated”, “Positive regulation of transcription from RNA polymerase II promoter”, “Cell proliferation”, and “Cell migration” in the BP category were highly enriched (**Figure 4F**). Intersection of the ChIP-Seq target genes with the above RNA-Seq DEGs revealed 38 overlapping genes, including 3 cell-cell adhesion genes (**Figures 4G, H**). These 3 genes were further analyzed by RT-qPCR (**Figure 4I**). The results showed that EphA2 is directly regulated by PTIP.

### PTIP Inhibits ESCC Cell Invasion and Migration Through Suppression of EphA2

Since PTIP was shown to directly regulate EphA2 expression in ESCC cells, we hypothesized that PTIP inhibits ESCC cell invasion and migration through transcriptional regulation of EphA2. Western blotting was performed to evaluate the expression of EphA2 in PTIP knockdown cells and further understand how PTIP regulates EphA2 expression (**Figure 5A**). Next, we assessed the correlation of EphA2 expression level and lymph node status in ESCC patients. Compare to non-invasive ESCC patients, EphA2 is highly expression in invasive patients (**Figures 5B–D**). In addition, pearson correlation coefficient indicates significant negative correlation between PTIP and EphA2 expression levels (**Figure 5E**). Rescue experiments show that knockdown of EphA2 could attenuate PTIP depletion promoted ESCC invasion (**Figures 5F–H**). These results showed that EphA2 was negatively correlated with the expression of PTIP, which is consistent with the sequencing results. Depletion of PTIP by shRNAs increased S897phosphorylation and decreased Y588 phosphorylation of EphA2 (**Figure 5A**), indicating that EphA2 enhance ESCC cell invasion through ligand-independent manner. In agreement with previous reports that EFNA1 promotes rapid turnover of phosphorylated EphA2. Overexpression of EFNA1 reduced the protein level of EphA2 in ESCC cells and inhibited the invasion of KYSE-150 cells. Although not significant, there was a similar trend in TE1 cells (**Figures S3a-f**).

**Figure 5:** PTIP inhibits ESCC cell invasion and migration through EphA2. **(A)** Western blotting analysis against PTIP, EphA2, pS897-EphA2, pY588-EphA2 in PTIP knockdown(shPTIP#1, shPTIP#2) and control (shCtrl) TE1 cells. **(B)** IHC score for EphA2 in ESCC tumor sections. Unpaired, two-tailed Student’s t-test; **P < 0.01. **(C)** Representative IHC images for EphA2 in ESCC tumor sections. Low EphA2 and high EphA2 groups were divided based on the EphA2 immunostaining intensity scores mentioned in method. Cut off for high and low EphA2 expression in ESCC was defined < or > 11. **(D)** Percentage of invasion and non-invasion in ESCC groups. The differences between rates were tested by χ2; *P < 0.05. **(E)** Comparative expression between PTIP and EphA2 in ESCC samples from **(B)** analyzed by Pearson correlation. **(F)** Knockdown efficiency of shRNAs targeting PTIP and EphA2 in TE1 cells as determined by qRT-PCR. One-way ANOVA; *P < 0.05,**P < 0.01, ***P < 0.001. **(G, H)** The effect of PTIP and EphA2 double knockdown on the invasiveness of TE1 cells. For invasion assay, six different microscopic fields (magnification, ×10) from at least three independent experiments were examined; Relative intensities of the fields were measured (n ≥3). Representative images and statistical plots are shown; Mean ± s.d. are given for three independent experiments. One-way ANOVA; ***P <0.001. **(I)** ChIP-seq density profiles for PTIP in TE1 cells. Gene models are shown below the density profiles. **(J, K)** ChIP-qPCR primer sets marked with arrows were designed to cover regions present within (EphA2) or outside (EphA2-NC) of the EphA2 gene **(C)**. ChIP-qPCR analyses of EphA2 binding **(D)**. Representative images and statistical plots are shown; Mean ± s.d. are given for three independent experiments. Unpaired, two-tailed Student’s t-test; **P < 0.01.

We next thoroughly analyzed the above ChIP-seq data and observed that a specific peak of PTIP overlapped in the intragenic regions of the EphA2 gene (**Figure 5I**). This result was verified by ChIP-qPCR using specific primers targeting the intron region of EphA2 (**Figures 5J, K**). Taken together, these data demonstrate that EphA2 is one of the downstream target genes of PTIP, indicating that PTIP plays a substantial role in ESCC through EphA2.

### PTIP Inhibits EphA2 Expression by Competing With Fosl2 for Binding to EphA2

To clarify the mechanism through which PTIP inhibits transcription of EphA2, we identified a series of PTIP highly enriched binding motifs using HOMER. The top 2 motifs of PTIP association were closely similar to the Fosl2(AP-1) and YY1 binding motifs (**Figure 6A**). Loss of function analysis shown that knockdown of Fosl2, but not YY1, increased EphA2 expression (**Figures 6B, C** and **Figure S4**). Next, cell invasion capability was robustly inhibited by depletion of Fosl2 in ESCC cells (**Figures 6D–G**). Indeed, ectopic expression of EphA2 partially rescued the hypo-invasive phenotype caused by knockdown of Fosl2 (**Figures 6H–M**).

**Figure 6:** PTIP inhibits EphA2 expression by competing with Fosl2 for binding to EphA2. **(A)** PTIP highly enriched binding motifs in bioPTIP ChIPseq were identified by HOMER. *P*-values are indicated within the boxes. **(B, C)** Western blot analysis of Fosl2 and EphA2 expression in Fosl2 knockdown (shFosl2#1, shFosl2#2) and control (shCtrl) TE1 **(B)** and KYSE-150 **(C)** cells. **(D–G)** The effect of Fosl2 knockdown on the invasiveness of TE1 **(D, E)** and KYSE-150 **(F, G)** cells. For invasion assay, six different microscopic fields (magnification, ×10) from at least three independent experiments were examined; Relative intensities of the fields were measured (n≥3). Representative images and statistical plots are shown; Mean ± s.d. are given for three independent experiments. One-way ANOVA; *P < 0.05; *P < 0.01; ***P < 0.001. **(H–M)** Western blot showing stable expression of Flag-EphA2 in shFosl2#1 TE1 cells **(H)** and KYSE-150 cells **(K)**. Overexpression EphA2 partially restored TE1 cells **(I, J)** and KYSE-150 cells **(L, M)** invasive ability, which attenuated by depletion of Fosl2. For invasion assay, six different microscopic fields (magnification, ×10) from at least three independent experiments were examined; Relative intensities of the fields were measured (n≥3). Representative images and statistical plots are shown; Mean ± s.d. are given for three independent experiments. One-way ANOVA; *P < 0.05; ***P < 0.001. **(N, O)** ChIP-qPCR analyses of the relationship between Fosl2 and PTIP in transcriptional regulation for EphA2. Mean ± s.d. are given for three independent experiments. Unpaired, two-tailed Student’s t-test; *P < 0.05.

Since PTIP and Fosl2 play opposing roles in regulating EphA2 and ESCC invasion, we hypothesized that PTIP and Fosl2 competitively occupy the cis-acting element of EphA2 to regulate EphA2 expression. To test this hypothesis, we next examined the relationship between Fosl2 and PTIP in the transcriptional regulation of EphA2. Indeed, when PTIP was knocked-down, the recruitment of Fosl2 to the EphA2 gene was dramatically increased compared to the control, and vice versa (**Figures 6N, O**). In a word, PTIP inhibited EphA2 expression by competing with Fosl2.

Our results provide evidence that PTIP competitively regulates EphA2 gene expression with Fosl2 to contribute to the invasiveness of ESCC cells. Our findings may offer potential therapeutic agents for the treatment of ESCC, such as small molecule modulators of PTIP or Fosl2.

## Discussion

A better understanding of the adhesion mechanisms responsible for tumor cell invasiveness is critical, as tumor cells with low adhesion may separate from each other. In this study, the mRNA profiles of lymph node metastasis–positive ESCC samples were compared to those without lymph node metastasis. Our results showed that PTIP was downregulated in ESCC samples positive for lymph node metastasis. Moreover, a significantly negative correlation was detected between PTIP expression and the lymph node metastasis status of ESCC patients. Western blotting and RNA-seq analyses showed that PTIP inhibited the expression of EphA2 in ESCC cells. More importantly, we found that PTIP knockdown could promote ESCC metastasis *in vivo* using a nude mouse xenograft model. In xenograft mouse tumor sections, the PTIP knockdown tumors showed increased lung metastasis compared with the control group. Taken together, these results indicate that PTIP inhibits lymph node metastasis in ESCC *in vivo*. Therefore, our findings reveal a novel PTIP function in which PTIP negatively regulates ESCC cell invasiveness by transcriptionally suppressing EphA2 gene expression.

During tumor progression, elevated levels of matrix metalloproteinases (MMPs) and decreased epithelial-mesenchymal transition (EMT) facilitate tumor cell invasion and metastasis (23, 24). It has been shown that mixed-lineage leukemia (MLL)-like complexes, including UTX, MLL4 and PTIP, play a significant role in cancer invasion and metastasis (25–27). In breast cancer, UTX (also known as KDM6A) and MLL4 enhance the invasion ability of breast cancer cells by promoting the expression of MMP family proteins (27). In our study, GO analysis showed that PTIP does not regulate the expression of MMP family proteins in ESCC cells, but regulates the expression of EMT-related genes. Further ChIP-seq results indicated that PTIP may indirectly regulate the expression of EMT-related genes.

In general, it is believed that PTIP acts as a transcription activator, through interaction with other MLL-like components such as UTX and MLL3 (16, 28, 29). Contrary to the prevailing perception that PTIP is solely a transcriptional activator, our study identified that it also functions as a repressor. These results are in agreement with findings by Fang et al. which showed that 52 genes were upregulated after PTIP knockdown in *Drosophila* Kc cells (29). In our study, we found that PTIP inhibited EphA2 expression by competing with Fosl2. Fosl2, a transcription factor of the activator protein-1 family, has been linked to cell adhesion, movement, invasion, metastasis, and cell growth (30). Overexpression of Fosl2 is associated with higher invasiveness in breast cancer (31). Indeed, our results showed that knockdown of Fosl2 significantly downregulated EphA2 expression and reduced the invasion ability of ESCC cells. Further investigation showed that PTIP and Fosl2 compete for binding to EphA2 cis-acting elements, thereby regulating gene expression and ultimately affecting the outcome of ESCC. It will be interesting to determine the relation between PTIP expression levels and overall survival in patients with ESCC.

Eph and ephrin are identified as contributors to tumor progression, hence they are considered to be attractive tumor markers and they are attractive targets for therapy. But so far, there are no drugs targeting Eph/ephrin family for medical use, because the interactions between Eph and ephrin are not specific and promiscuous (8). Therefore, targeting the upstream regulators of EphA2 may provide additional targets for cancers. Previous studies have shown that the expression of EphA2 is regulated by multiple elements in human cancers (32–35). In HCC cells, testicular nuclear receptor 4 (TR_4_) directly binds to the TR_4_-response element located on the 5’ promoter of EphA2, suppressing its transcription, and subsequently inhibiting HCC cell migration/invasion (32). Another study showed that the KRAS-driven MAPK and RalGDS-RalA signaling pathways promote EphA2 expression in colorectal (36). Moreover, EphA2 was also downregulated by miR-302b in gastric cancer. In this study, we revealed that EphA2 is regulated by PTIP and Fosl2 in ESCC. Targeting PTIP or Fosl2 may offer a route to circumvent the limitation of Eph/ephrin in drug development. Further preclinical evaluation of targeting PTIP and Fosl2 as a strategy to block tumor metastasis is therefore warranted. Similarly, further details of how PTIP is upregulated in ESCC cells need to be determined.

## Data Availability Statement

The datasets presented in this study can be found in online repositories. The name of the repository and accession numbers can be found below: National Center for Biotechnology Information (NCBI) Sequence Read Archive (SRA), https://www.ncbi.nlm.nih.gov/sra/, SRR13089664 to SRR13089679.

## Ethics Statement

The studies involving human participants were reviewed and approved by the Huaian No.1 People’s Hospitals’ Ethics Committee. The patients/participants provided their written informed consent to participate in this study. The animal study was reviewed and approved by the Animal Experimentation Ethics Committee of Huai’an First People’s Hospital.

## Author Contributions

XH performed experiments, analyzed, and interpreted data. YZhu performed experiments and analyzed data. LS, YZhou, and HG helped perform the experiments. WZ assisted with the Immunohistochemistry. LP, KH, YY, CJ, and JX collected and performed experiments using human CML samples. CZ designed the research, wrote the paper and provided the funding. LD designed the research and supervised the experiments. All authors contributed to the article and approved the submitted version.

## Funding

This work was supported by the National Natural Science Foundation of China (81500128), the Entrepreneurship and Innovation Project in Jiangsu Province and the Innovative Capacity-Building Plan in Huai’an (HAP201702).

## Conflict of Interest

The authors declare that the research was conducted in the absence of any commercial or financial relationships that could be construed as a potential conflict of interest.

## Supplementary Material

Supplementary Figure 1 Depletion of PTIP do not alter ESCC cell survival, EC-matrix adhesion and morphology. **(a)** Representative FACS dotplots of YF647A-AnnexinV/PI staining used to assess apoptosis after knockdown of PTIP using two independent shRNAs targeting PTIP in the TE1 and KYSE-150 cell lines. **(b)** The rates of apoptosis in shCtrl versus shPTIP ESCC cells were determined by FACS. Mean ± s.d. are given for three in-dependent experiments. **(c)** Knockdown of PTIP did not significantly alter ESCC cell adhesion to collagen I. One-way ANOVA; **P* < 0.05. **(d)** Representative images of phalloidin staining in ESCC cells.

Supplementary Figure 2 PTIP overexpression in ESCC cells did not significantly inhibit cell invasion. **(a-f)** Western blot showing stable expression of Flag-PTIP in TE1 cells **(a)** and KYSE-150 cells **(d)**. Overexpression PTIP did not inhibit TE1 cells **(b,c)** and KYSE-150 cells **(e,f)** invasion. For invasion assay, six different microscopic fields (magnification, ×10) from at least three independent experiments were examined; Relative intensities of the fields were measured (n≥3). Representative images and statistical plots are shown; Mean ± s.d. are given for three independent experiments. One-way ANOVA; n.s., not significant.

Supplementary Figure 3 EFNA1 overexpression in ESCC cells decreased EphA2 expression level and inhibit cell invasion in KYSE-150. **(a-f)** Western blot showing stable expression of Flag-EFNA1 in TE1 cells **(a)** and KYSE-150 cells **(d)** decreased EphA2 expression. Overexpression EFNA1 did not inhibit TE1 cells invasion **(b,c)**, but not in KYSE-150 cells **(e,f)**. For invasion assay, six different microscopic fields (magnification, ×10) from at least three independent experiments were examined; Relative intensities of the fields were measured (n≥3). Representative images and statistical plots are shown; Mean ± s.d. are given for three independent experiments. One-way ANOVA; n.s., not significant; ***P* < 0.01.

Supplementary Figure 4 Depletion of YY1 did not increase EphA2 expression in ESCC cells. Western blotting analysis against EphA2, YY1 and GAPDH in YY1 knockdown(shYY1#1, shYY1#2) and control (shCtrl) TE1 cells.
